# Simulation Training Auxiliary Model Based on Neural Network and Virtual Reality Technology

**DOI:** 10.1155/2022/2636877

**Published:** 2022-07-01

**Authors:** Wei Liu

**Affiliations:** Guangzhou Panyu Polytechnic, Guangzhou 511400, China

## Abstract

Training simulators have been gradually evolving in the direction of software, virtualization, networking, and multiplatform in recent years, with the continuous development of hardware and software technologies, particularly the maturity of VR (Virtual Reality) related technologies. The network intrusion program allows remote hackers to take control of the system, posing a serious threat to the network and computer security. As a result, this paper proposes a VR-based ID (intrusion detection) simulation training system. This paper proposes an ID model based on CNN (Convolutional Neural Networks) and LSTM to address these issues (Long Short-term Memory Networks). This model oversamples data from unbalanced data sets, reducing the difference in category data and thus improving the ID model's performance and existing detection methods to compensate for the flaw. 3DSMAX technology is used to simulate the process visualization scene, as well as some key equipment models and signal transmission simulations, during the system design and implementation process. The experimental results show that CNN LSTM outperforms BP, and the overall evaluation index *F*1 has significantly improved, particularly the *F*1 index of D4. CNN LSTM outperforms GA (genetic algorithm) by 12.75 percent and BP by 14.07 percent. The system essentially accomplishes the anticipated simulation training goal, and the simulation training effect is impressive.

## 1. Introduction

As a means of information transmission and communication, virtual reality technology can intuitively and realistically provide students with visual information such as the structure, size, working principle, and assembly process of equipment, allowing them to observe the team in a virtual environment. The working process and direct operation of each component help students understand and perceive tasks more effectively. Virtual reality is a new technology. Its goal is to make the information system as user-friendly as possible, to improve the direct interaction between users and data, and to make human-computer interaction more convenient and humanized [1]. The simulation training system based on VR technology has low cost, high versatility, easy upgrade, and easy maintenance, among other features, and is particularly well suited to the primary training of students' operation skills.

Network security technology has become a key technology of computer networks. ID (intrusion detection) is considered the second security door behind the firewall. It can monitor the network without affecting the network performance, provide real-time protection against internal attacks, external attacks, and improper operations, and greatly improve network security [2]. An efficient ID system can provide security for the computer system, network system, and even the whole information system and prevent huge economic losses. Wang et al. have studied and implemented a real-time ID system model, which is based on the profile of user behavior characteristics and uses statistical methods to describe the behavior of system subjects relative to system objects [3]. Riyaz and Ganapathy adopted a recursive network and combined it with traditional expert system for ID [4]. Esmeir and Markovitch proposed an anomaly detection algorithm based on a one-dimensional self-organizing feature mapping network [5]. Alkadi et al. introduced information retrieval technology into ID. However, some algorithms are not practical, such as expert methods [6], and some algorithms are still in the experimental research stage, such as immunological methods and neural networks.

By examining the current state of information security, we can see that traditional security technology is unable to fully guarantee network security, and the existing ID system has numerous flaws. As a result, the development of identification technology must meet higher requirements in order to protect network security. The system may be attacked, according to the current security situation. If the system is attacked, further losses can be avoided if the attack is detected as quickly as possible, even in real time. In this regard, identity verification is critical for establishing a security system capable of compensating for the shortcomings of traditional security measures. This document develops an ID simulation training system using VR technology based on the ID process and the use of 3DSMAX software. Simultaneously, it can effectively solve students' learning and training problems, improve the efficiency of students' knowledge absorption, master skills, and improve the effectiveness of education and training. This paper contains the following innovations:

1. In this paper, a simulation training system is established, and the virtual training scene is constructed and optimized by 3D modeling and 3DSMAX rendering software. Finally, the interactive settings of die-cutting, paper, and die-cutting actions are made by VR software, and the training interaction of virtual ID is realized.
2. This paper presents an ID detection model based on a neural network. This model can extract the local features of data in the network by using CNN's deep feature learning [7, 8], which can improve the accuracy of ID and reduce the false alarm rate.

This paper has the following organizational structure: The first chapter discusses the research's background and significance before moving on to the paper's main work. The second chapter focuses on the technologies that are needed to implement the simulation training system. The research's concrete methods and implementation are presented in the third chapter. The superiority and feasibility of this research model are confirmed in the fourth chapter. The summary of the full text appears in the fifth chapter.

## 2. Related Work

### 2.1. ID System Research

After analyzing the characteristics of the traffic flowing through the network, ID can analyze the user's behavior to see if it is malicious, which is an active tracking behavior. From here on, ID has entered the development stage of network detection.

Fan et al. adopted a multilevel hierarchical ID method based on GA (genetic algorithm) to solve the problems of a single-level ID system [9]. Ghosh et al. proposed a method of constructing an ID system with a decision tree, which can identify unknown attacks in the network [10]. Alotaibi and Alotaibi proposed an abnormal traffic detection method based on a deep neural network, which can identify the normal or abnormal connections in the network, and the detection effect is good [11]. Kumar et al. proposed a deep neural network ID system based on context LSTM (Long Short-term Memory Networks) [12]. Firstly, the original data is obtained by social media on the internet, from which the push-level bots are detected, and then the context features are extracted and detected by LSTM. However, this method is only suitable for the detection of specific bots.

Kim et al. used a standard BP network to train and recognize the formed user behavior feature vectors [13]. Choobdar et al. used two different statistical analysis detection techniques to detect the abnormal behavior of the system [14]. Tian et al. used comprehensive traffic monitoring to find anomalies, combined with geographic information to show the location of intrusion events and applied the corresponding relationship between intrusion and vulnerability to give the risk analysis results between intrusion threats and asset vulnerability so as to effectively manage security events and timely handle and respond [15]. Rezaei and Liu applied the immune principle to the field of distributed ID [16].

### 2.2. VR Technology Research

In recent years, with the continuous development of computer hardware and software, new technology has developed rapidly-VR. It is an ideal man-machine interface between VR computers and users. VR system has three important characteristics: immersion, interactivity, and imagination. VR technology has a wide range of potential applications, such as national defense, architectural design, industrial design, training, medical treatment, and other fields.

With the help of specially designed sensors, users can interact with 3D images and manipulate virtual objects so that users can perceive the virtual environment equivalent to the real world [17]. Xue et al. further simplified it into a computer program that can present a simulated world [18]. It can be defined as a highly interactive three-dimensional digital media environment. Users can intuitively experience the simulated environment and get multisensory feedback such as hearing, touch, and vision. Wang and Zhu think that good spatial audio not only makes users deeply immersed in a virtual environment but also is an important channel for users to obtain environmental information [19]. Yong proposed an optical mapping near-eye 3D display method for wearable devices, the core of which is to adjust the eyes to the same distance as a binocular stereo vision to relieve eye fatigue and discomfort [20]. Compared with previous methods, this monitor has outstanding advantages in adaptability, dynamic range of images, and refresh rate.

It is a somatosensory interaction technology to interact with the virtual environment in a noncontact way through physical natural behaviors such as actions, sounds, or expressions. Foreign scholars generally believe that somatosensory interaction technology is a key component of VR and plays an important role in VR training. Yang et al. put forward a soft motion sensing device for measuring lower limb joint motion, which can effectively improve the shortcomings of the prior art in mobility and wear resistance [21]. Xia and Qi proved that distributed VR system can build a 3D collaboration environment for distributed users to interact with each other and complete various collaboration tasks [22]. Distributed VR system conforms to the new demands of the times, promotes communication and collaboration among users, and their application potential needs to be explored more. Bai et al. are committed to improving the user experience of VR devices, suggesting that a multiuser VR environment and wireless connection should be considered in future VR devices [23].

## 3. Methodology

### 3.1. ID Model Design

The algorithm used by the ID system has a direct impact on detection efficiency and accuracy. Pattern matching is now one of the most widely used detection methods and mechanisms in the field of identification. The next step in this concept is to define the pattern of existing problems. Then look for event data that corresponds to the pattern. Anomaly detection and production ID systems frequently employ statistics. Statistics is a relatively mature ID method that allows the ID system to learn the subjects' daily behavior and identify those activities that statistically differ from normal activities as abnormal. Because of the immune system's unique capabilities, an ID system based on immunological methods offers numerous benefits, including diversity, fault tolerance, distribution, dynamics, self-management, and adaptability.

The neural network has the ability of self-adaptation, self-organization, and self-learning. It can deal with some problems with complex environmental information and unknown background knowledge, which makes the samples have big defects and deficiencies [2]. From the perspective of pattern recognition, an ID system can use a neural network to extract pattern features from user behavior and then create profiles of user behavior features. In a word, the introduction of the neural network into the ID system can solve the dynamic characteristics of user behavior and the difficulty of accurate detection caused by incomplete and uncertain search data. The attack behavior in the network is not completed at a single point in time but will be sent continuously over a period of time. By analyzing the correlation performance of the time series before and after the network data, the intrusion behavior can be best detected. In this paper, an ID model combining CNN (Progressive Neural Network) and LSTM (Long Short-term Memory Networks) is proposed, and the loss function is optimized to improve the ID accuracy and reduce the false alarm rate. The ID is shown in Figure 1.

In this model, CNN is first used to extract depth local features in order to effectively extract sample data, and then LSTM is used to learn and extract correlation features between continuous data in both positive and negative directions. Finally, the softmax layer is used for classification, and the Focal Loss function is used to optimize the model. The model takes into account the temporal and spatial correlation of intrusion data and can extract unknown features and internal dependencies between data, lowering false alarm rates and improving detection effectiveness.

The role of the ID model based on deep learning is to divide the emerging abnormal data traffic into a group of known attack types according to their function or behavior. In the actual detection process, it is often necessary to preprocess the samples, including digitization, normalization, data equalization, and other operations, so as to make the data conform to the input format of the detection algorithm.

Select to keep the useful information in the memory cell, discard the unnecessary information, and normalize the value by activating the function. The specific calculation formula is shown as follows:

(1) $$\begin{array}{c} f_{t}=\sigma \left(W_{f}\cdot \left[h_{t-1},x_{t}\right]+b_{f}\right). \end{array}$$

*σ* is the sigmoid function. At *t* − 1 time, the output vector of the hidden layer is expressed as *h*(*t* − 1), at *t* time, the input vector is expressed as *x*_*t*_, and in *f* state, the weight matrix of *x*_*t*_ is expressed as *W*_*f*_, and *b*_*f*_ is offset.

In the ID model designed in this paper, there is only one full connection layer, and the upper layer information is integrated and transmitted to LSTM. The output calculation formula of neurons in the whole layer is shown in the following:

(2) $$\begin{array}{c} y_{j}^{l}=\sum_{i}w_{\text{ij}}^{l}*x_{i}^{l-1}+b_{j}^{l}, \end{array}$$

where *w*_ij_^*l*^ represents the connection weight; *x*_*i*_^*l*−1^ is the *i* th eigenvalue of the eigenvector in layer *l* − 1; *b*_*j*_^*l*^ represents the offset value; *y*_*j*_^*l*^ is the calculated output of the *j*-th neuron in layer *l*.

Input the sample vector into the *X* competition layer, calculate the Euclidean distance between the sample point and the subcategory, and find the most suitable subcategory to belong to the following:

(3) $$\begin{array}{c} d\left(X,W_{c}\right)=\min\left\{d\left(X,W_{i}\right)\right\}\;i=1,2,\ldots ,R, \end{array}$$

where *W*_*c*_ represents the initial weight of the network, *d*(*X*, *W*_*c*_) represents the distance between the *i* th input sample and the subcategory, and *W*_*i*_ represents the subcategory after winning the competition.

*x*_ij_ is set as training data, which contains data elements with large variation. The goal is to make the variation between elements less than 1. First calculate the average of all elements in *X*:

(4) $$\begin{array}{c} p_{0}=\frac{1}{m*n}\sum_{i=1}^{n}\sum_{j=1}^{n}x_{\text{ij}}. \end{array}$$

Among them, *i*=1,2,…, *m*; *j*=1,2,…, *n*.

Then, through a mapping function, the numerical values are mapped to each subinterval to be quantified so as to achieve the goal of normalization. The normalization method used here is linear normalization, and the expression is as shown in the following formula:

(5) $$\begin{array}{c} y=\frac{x-\text{Min Value}}{\text{Max Value}-\text{Min Value}}, \end{array}$$

where *x*, *y* is the value before and after conversion, and Max Value, Min Value is the maximum and minimum value of the sample.

If the output is close to [0, 1], it is assumed that an intrusion has occurred, and the control center should be notified and appropriate measures taken. If the intrusion is new, the neural network should be investigated, retrained, the weights corrected, and the network's performance improved. Distributed object technology, software agent technology, and mobile code technology are all combined in mobile agent technology. It is a brand new computing technique for dealing with complex, dynamic, and distributed intelligent applications. The concept of distributed computing has been greatly expanded by the addition of intelligent functions and mobile creativity. Artificial intelligence combined with distributed computing is likely to become a key component of intelligent distributed computing.  Figure 2 is the flow chart of mobile agent task analysis.

The scheduling manager is the core component of the mobile agent service environment. Assign all kinds of services required for normal mobile agent operation to the corresponding submodules, including setting the mobile agent execution environment, starting services, etc. In addition, it is also responsible for coordinating the cooperation among submodules to ensure their normal operation. Static agent mainly completes the interaction between agent scheduling manager and front-end agent.

### 3.2. Scene Modeling

One of the keys to building a high-fidelity virtual scene is to use 3D modeling technology and modeling software to present a scene almost identical to the real environment on the computer. Realistic virtual ID model is the basis of designing a virtual die-cutting training system as a visual, interactive, and realistic simulation training scene of die-cutting equipment. Virtual identity recognition is an important core part of the virtual simulation training system. Because these devices require high precision, this paper uses Solidworks to build parametric models of these devices and then imports them into 3DsMax for rendering, which can not only ensure the model precision but also ensure the fidelity.

Unique training is done by plane animation. An image is an original hand-drawn painting, and Photoshop is used to perform the effects of the image, such as color correction, motion processing, and stereo effects. The transition and continuity of actions are completed through key frames to ensure the accuracy and consistency of actions. It should be noted that when modeling in 3D Studio Max, the material must use standard material or multisubobject material and use the default scanline renderer. All the sizes of the maps are set according to the pixel of 2 to the *n* power, so as to reduce the memory overhead and improve the fluency of the software.

For a surface *S*, suppose we need to paste texture lines on the surface. First, we need to find out the relationship between space *A* and *B*. Let the radius of the surface *S* be *R* , and the chord height PF=*h* be OP=*R* − *h*; Make AB=*x*, so we can get the following relationship:

(6) $$\begin{array}{c} \frac{R}{R+x}=\frac{R-h}{R}. \end{array}$$

After simplification, you get the following:

(7) $$\begin{array}{c} x=\frac{\text{hR}}{h-R}. \end{array}$$

There are

(8) $$\begin{array}{c} {\left(s-x^{*}\right)}^{2}+{\left(t-y^{*}\right)}^{2}+z^{*}={\left(\frac{\text{hR}}{h-R}\right)}^{2}. \end{array}$$

Then the *B*(*x*^*∗*^, *y*^*∗*^, *z*^*∗*^) on the curved surface corresponds to the *A*(*s*, *t*) on the texture pattern one by one, and similarly, other surfaces on the curved surface also have this corresponding relationship.

So you can get the following:

(9) $$\begin{array}{c} \sin\;\theta =\frac{\left|\text{AB}\right|}{\left|A^{*}B^{*}\right|}=\frac{\text{am}+\text{bn}+\text{cp}}{\sqrt{{\left(x_{1}^{*}-x_{2}^{*}\right)}^{2}{\left(y_{1}^{*}-y_{2}^{*}\right)}^{2}{\left(z_{1}^{*}-z_{2}^{*}\right)}^{2}}}. \end{array}$$

After the above transformation, the texture space coordinate (*x*, *y*) and the concave-convex model mapping area coordinate (*x*^*∗*^, *y*^*∗*^, *z*^*∗*^) can form a one-to-one correspondence relationship so as to better realize concave-convex model mapping.

The color and properties of materials should be as close to real objects as possible to improve the fidelity of virtual scenes. Material Editor and Material/Map Browser tools are included in 3ds Max. You can choose different types of shading for objects, use different material components, and enhance materials with maps to make them look more realistic in light and environment in the Material Editor. To achieve the desired effect, we simply need to set and adjust the parameters of the particle system according to the characteristics of special effects during the development process. The time it takes to write and develop code can be cut in half while achieving special effects, and good results have been obtained [12].

### 3.3. Realization of Interactive Effect of Virtual Scene

As an important part of the network attack and defense training system, ID simulation training system mainly includes four main subsystems, as shown in Figure 3. The subsystem uses the database SQLServer database (the database name is net_fight) to store data. As the data storage center of the whole education and training system, the input subsystem is the general part of the whole education and training system and undertakes various input and output functions.

In this virtual simulation training system, there are many virtual scenes that need to interact with each other in order to realize the real representation of identity. Paper feeding includes two parts: paper feeding and paper discharging after die-cutting. Paper movement is set interactively with the path node, and the path node can move or rotate its parent node. In its property box, you can enter the moving position and direction of the paper at each time point to make the paper move along a certain path. Use the place node to complete the previous movement. When the start button is pressed, the template immediately rises. A user-defined function node can be described using a Script node. You must define a field list, event input and output, and what to do with these operations in this function node. The student users enter the Train system and begin attack training after the teacher has been set up. The student's attack is successful if the attack condition matches successfully; if the condition fails, the student immediately enters the temporary result and starts over. The attack subsystem's network intrusion function simulation module also sends interface information to the input-output subsystem, which saves the final information in the result data table.

Attack sequence table attack_state table stores information about students' attacks and Source_IP field indicates the IP address of the attacker. Server setup simulation includes verification code setting, password setting, server name setting, online prompt setting of the destination host and sending to mailbox, etc. When “student_state” = “1,” the target IP is online; when “student_server” = “1,” the target host has an intrusion server installed on the network.

## 4. Experiment and Results

In the experiment, 100,216 randomly selected and preprocessed data blocks are used as training sets for model training, and 4,227 randomly selected data blocks are used as test sets for performance testing. After numerical processing in data preprocessing, the single record in the set is finally changed from the original 40-dimensional feature vector to the 120-dimensional binary feature vector. Therefore, the model input in this document is a numerical array with a fixed size of 1*∗*120. In this paper, the loss function parameter *α*=0.2, *γ*=3, which has been verified by the existing experiments, has been used for many experiments. Recall rate and false alarm rate are used as performance evaluation criteria. Experimental results are shown in Table 1.

The experimental results in the above table are displayed visually by charts, as shown in Figures 4 and 5.

According to the analysis of Figure 4, the recall rate first rises and then falls with the increase of the convolution kernel, and the difference is obvious. When the convolution kernel size is 5 and the number of hidden layer ganglia is 30, the recall rate reaches the maximum value. According to the false alarm rate in Figure 5, when the convolution kernel size is 5 and the number of hidden layer nodes is 30, the false alarm rate is the lowest, and the larger the convolution kernel, the greater the error. Considering these two results, the optimal combination scheme is selected. In this paper, the size of the convolution kernel is set to 5, and the number of ganglion points in the hidden layer is set to 30.

In this paper, the experimental results of *F*1 overall evaluation indexes of three models on five data types are also given to verify the classification effect of the models on a few classes. The results are shown in Figure 6.

It can be seen that CNN_LSTM has more advantages than BP, and the overall evaluation index *F*1 has improved a lot. The *F*1 index of D_4 CNN_LSTM is 12.75% higher than GA and 14.07% higher than BP. The results verify the effectiveness of the data processed by oversampling method and the model trained by the Focal Loss function on unbalanced data sets.

The false positive and false negative rates have a direct impact on whether the system can be used in real-world situations. Although the neural model ID system can detect new types of intrusions that were previously unknown, it cannot completely eliminate the problem of false positives and false negatives. Establish the object's abnormal activity pattern, and by observing the proximity between current activity and the abnormal activity pattern, detect the same type of intrusion behaviour. The neural network is used for reverse learning when the rule system detects the intrusion, and the neural network ID is used at other times. When an intrusion occurs, the double detection system can reduce false alarms.

The training data is input into CNN_LSTM for training, and the actual output simout is compared with the expected output simt, and the detection result of the whole neural network is obtained. Make *θ*_1_=*θ*_2_, then take different values, and test with CNN_LSTM, which has been trained before. The experimental results are shown in Table 2:

It can be seen from the above table that the higher the threshold, the higher the false alarm rate and the lower the false alarm rate, while the lower the threshold, the lower the false alarm rate and the higher the false alarm rate, which is a contradictory relationship. If the false alarm rate is low, the false alarm rate will increase. If the false alarm rate is low, the false alarm rate will increase. Therefore, users can set appropriate thresholds according to their own needs so that the ID system can achieve the best detection performance.

Learning network intrusion takes place in virtual machines, and it consists of two parts: learning the statistical characteristics of normal users during operation and learning intrusion. When the system is in place, ordinary users' operation learning is completed, and many existing research results can be used as a reference. The virtual machine adapts the running parameters, extracts statistical data from the data packet conversion expert database, adjusts the input, and performs network learning based on the situation, determining if the learning is complete in light of the convergence situation and updating the neural network detection model. Following the completion of the neural network's learning and training, the pattern discrimination work is converted into a numerical operation that can be executed at high speed on a computer, resulting in an efficient parallel nonlinear dynamic processing system that can meet real-time processing requirements. The false alarm should theoretically be a subset of two independent systems for dual-system operation, which can greatly reduce the false alarm rate. New intrusion rules can be obtained through log analysis, and rule detection rules can be added to the rule detection system to make it more perfect.

The efficiency of the pattern matching algorithm is determined by three factors: text length, pattern length, and alphabet size. Because no pattern matching algorithm is optimal under all conditions, the purpose of the experiment is to test the performance of each algorithm when the above factors are modified.  Figure 7 shows the execution time comparison of the three algorithms.

It can be seen from Figure 7 that the execution speed of CNN_LSTM is slightly faster than that of reference [18] algorithm and reference [20] algorithm. When the protected system is very important and the system manager needs to constantly correct the rules, it is necessary to collect the information of intruders, constantly improve and optimize the system, and transfer intruders to dedicated servers. The most common alarm and notification method provided by the ID system is the screen alarm. When the ID system is installed, this alarm information will appear on the ID system console or other user-configured systems. They only process local data and only return the results to the control center, so there is no delay caused by network transmission, and the bandwidth occupied by original data transmission can be saved. Another advantage of processing data on each node is that it can be processed in parallel, which will improve the detection speed.

It can be found from Figure 8 that the total number of character comparisons of CNN_LSTM is always less than that of reference [18] algorithm and reference [20] algorithm, no matter how the pattern string length and text string length change.

This advantage becomes more apparent as the pattern string length increases. Because the length of a pattern string in an ID system is usually between 20 and 30, the CNN LSTM algorithm has some utility in an ID system. Finally, when compared to the first two algorithms, the CNN LSTM algorithm has a shorter execution time. As a result, each algorithm corresponds to a specific number of simple operations, and the more times an algorithm is executed, the longer the execution time. As a result, the number of simple operations included in an algorithm is commonly referred to as the algorithm's time complexity, which is used to assess the algorithm's runtime or computational performance. We must set up a neural network module for unknown intrusion behavior to judge whether it is an attack behavior through repeated training of unknown behavior. The data from the data processing module cannot be sent directly to the neural network for identification; instead, it must be preprocessed to obtain data that meets the requirements. Then, the next time the system is used, the uncertain “behaviour” judged in the first job is updated to the known attack information, and the alarm module is directly used to give an alarm, eliminating the need to enter the neural network and greatly improving the ID system's efficiency and practicability.

## 5. Conclusions

In this paper, VR technology is applied to ID simulation training, and an ID simulation training system is designed and implemented using the 3DSMAX software development platform. Through the combination of virtual and real simulation, the problem is that network intrusion software has special functions and powerful remote control functions, and it is difficult to achieve good simulation results while ensuring network security is overcome. File management, registration, etc., and safely complete functions such as table management, video monitoring, screen control, etc. In this paper, a detection method combining CNN and LSTM is proposed. Softmax is used for classification, and the Focal Loss function is used on the Softmax layer to optimize the model. This method comprehensively considers the temporal and spatial correlation of intrusion data and can extract unknown features and internal dependencies between data, improve the ID accuracy, and reduce the false alarm rate. The experimental results show that CNN_LSTM has more advantages than BP, and the overall evaluation rate *F*1 has been greatly improved. The *F*1 rate of D_4 CNN_LSTM is 12.75% higher than GA and 14.07% higher than BP. The results verify the effectiveness of the data processed by oversampling method and the model trained by the Focal Loss function on unbalanced data sets.

## Figures and Tables

**Figure 1:** ID structure.

**Figure 2:** Flow chart of mobile agent task solving.

**Figure 3:** System structure.

**Figure 4:** Influence of convolution kernel size and number of hidden layer nodes on recall.

**Figure 5:** Influence of convolution kernel size and numb of hidden layer node on false alarm rate.

**Figure 6:** The *F*1 values of three types of detection for different categories.

**Figure 7:** Comparison of the execution time of three algorithms.

**Figure 8:** Total character comparison times of various algorithms.

**Table 1:** Influence of the number of hidden layer nodes on performance.

Convolutionkernel size	Number of hiddenlayer nodes	Precision(%)	False alarmrate (%)
1	10	93.31	2.17
1	30	94.15	2.26
1	60	93.36	2.54
5	10	93.01	2.24
5	30	94.41	2.01
5	60	93.96	2.21
8	10	93.02	2.23
8	30	92.28	2.63
8	60	94.65	2.51
13	10	94.55	2.66
13	30	93.38	2.71
13	60	92.16	2.89

**Table 2:** Experimental results with different thresholds.

Threshold value	False alarm rate	False alarm rate
0.2	0.0061	0.22
0.4	0.0073	0.26
0.6	0.0082	0.12
0.8	0.021	0.086

## Data Availability

The data used to support the findings of this study are available from the author upon request.
